# Prioritizing and Overcoming Barriers to e-Health Use among Elderly People: Implementation of the Analytical Hierarchical Process (AHP)

**DOI:** 10.1155/2022/7852806

**Published:** 2022-04-11

**Authors:** Ayesha Mumtaz

**Affiliations:** ^1^School of Public Administration, Hangzhou Normal University, Hangzhou, China; ^2^College of Public Administration, Zhejiang University, Hangzhou, China

## Abstract

Rise in the aging population brings new challenges to modern societies. Old age is associated with several morbidities and usual issues related to health. Therefore, the provision of healthy and timely care has become the dire need to maintain their quality of life and wellbeing. The evolution of the e-health care system put pressure on societies to implement it successfully to ensure a safe and prompt provision of care services to the most vulnerable population successfully. Therefore, the provision and implementation of the e-health care system is a challenge for the health industry in terms of multi-objective decision-making. Multicriteria decision-making is a generalizable approach to making decisions with dependence and feedback and is known as an effective tool in decision-making processes, particularly in the healthcare sector. The present study aims to present an e-healthcare framework by identifying and prioritizing potential barriers towards the use of e-health by the elderly population. The analytical hierarchy process approach is adopted to calculate weights of identified potential barriers, respectively, and then rank them based on their degree of significance. The findings show that health and the ability-related barrier is ranked highest, followed by socio-environmental and attitudinal barriers. This research contributes to healthcare decision-making regarding e-health usage by implementing MCDA techniques. Our study will assist the public health practitioners and policymakers in drawing decisions on the best strategy to minimize the risks in using the e-healthcare system by the aging population, which significantly contributes to the smart healthcare system.

## 1. Introduction

The world enters a new stage of development under the pressure of an aging population. Globally, the elderly population aged 65 exceeded 703 million [1]. The number of older persons is projected to double to 1.5 billion in 2050. Nevertheless, the awareness about the aging challenge is sharp. While this sudden trend in the aging population towards old age is already prominent in high-income countries, for instance, in Japan, where 30% of the total population is already over 60 years old. Thus, the trends in the aging population in developing and, middle- or low-income countries are also in transition. It is being estimated that two-thirds of the population in the world aged 60 or over will live in low- and middle-income countries in 2050 [1]. Under these circumstances, the issues of elderly care attract wide attention from scholars and policymakers, resulting in a large amount of research done in this field.

The use of e-health care systems by elderly people has already become a common trend worldwide [2]. To ensure the promotion of a healthy society, the need for modern care services has become a dire need of age, which is evidenced by the extensive e-healthcare requirements adopted during the recent Covid-19 pandemic [3]. To improve the healthcare system for elderly people, most of the developing countries are also growing their smart care industries and modernizing their health care settings [4]. The elderly health care industry is shifting from traditional family care to the smart care system to facilitate the elderly and their caregivers. Efficient use of technology is especially imperative in creating a more independent and supportive living environment for older people [5], stimulate their physical and psychosocial wellbeing, and enables them to feel more independent at their daily chores [6], interact with their families and friends [7], and to contribute to the elderly healthcare sector. The usage and adoption of e-health technology have become an established research area targeting at investigating the influencing factors affecting the usage of e-health [8–10]. Research in this area mainly focused on developed countries [8, 11], while the experiences of developing countries are rarely discussed, particularly addressing the e-health care industry.

Based on this, including the importance of e-healthcare in the present era, the adhesion of elderly people to e-health acceptance, and the recognition that elderly people in Pakistan are less optimistic about using technology, we were motivated to investigate this research gap. By keeping in view the vulnerable situation of the e-health care industry for the elderly, and the lack of research in this area, the researchers aimed to provide a foundation by conducting a pioneer research study. The use of e-health among the elderly is not a very common trend in Pakistan, and there is a lack of research in gerontechnology. However, the majority of the cities in Pakistan have telecommunication links and 531,787 broadband connections are provided to more than 1800 cities and 400 cities have the facility of fiber optics in Pakistan, which gives them access to universal healthcare information to elderly and their families. There are organizational barriers, lack of the interest of stakeholders, less motivation from friends and family, anxiety to use and adopt technology and also healthcare professionals do not play their role to promote the use of technology in Pakistan [12]. Given the scarcity of research on the technology usage behavior of elderly people in Pakistan, we were motivated to identify the barriers that influence the e-health usage behavior of elderly people.

Initially, a review of previous literature on the use of technology among the elderly has been conducted for this purpose. Further, a set of specific factors in different domains were identified based on the previous research findings. By answering the research question and objective, the subsequent contributions are proposed. The main contribution of this research to academia is the identification of the barriers to e-health care usage and detailed review of existing technology acceptance literature. Research on gerontechnology is scarce and our study intends to provide a detailed examination of the barriers to the usage of e-healthcare. Furthermore, for the business sector, our research identifies factors to consider when promoting e-healthcare products and services. The elderly smart care industry is developing very fast in the whole world. Thus, such research is critical for the elderly smart care industry, which is considering developing smart technology products for its elderly consumer market segment. Moreover, the methodological contribution of this study also provides new insights regarding e-healthcare, with the application of AHP as a premise to identify the less and more potential criteria for researchers and decision-makers.

To help readers understand the context, the following section identifies the various barriers identified by previous research studies as well as models for using e-healthcare technology. The previous researches have highlighted some basic factors which provided a foundation to identify the critical factors pertinent to e-health use. However, there is a lack of research in concepts relevant to this study which are all aligned to provide a methodological base to this study. The primary research question addressed in this study is “what are the potential barriers affecting the use of the e-healthcare system by elderly people, and how can these barriers be prioritized pertinent to the old age group”? Based on the review of the previous studies, 13 age-specific barriers were identified and categorized into main three categories. The literature review method is used in this study to identify the barriers of e-healthcare use. Next, Analytical hierarchal process (AHP) decision-making analysis is used to allocate weights to the main and sub-barriers by using the pairwise matrix technique [13]. The study includes the MCDM methodology, findings, discussion, and conclusion in subsequent sections.

## 2. Literature Review

Previous research studies mainly based on the intention or motivation to use technology [5, 14, 15], whereas, the research is scarce addressed the question of why older adults fail to use technology and what are the potential barriers? In this study, e-health system is defined as the digital or electronic healthcare products and services which increase the social independence and participation of elderly people relatively for health purposes [16]. The few researches that already have sought to investigate the reasons for using or not using technology have yielded somewhat contradictory results [17]. Although researchers revealed that older people have a positive attitude towards technology [5, 18], hence they are less likely to use those technologies due to some barriers as compared to young adults [19–21]. There are several reasons revealed by different studies for the use or nonuse of technology by elderly people. A study revealed that elderly people have negative attitudes towards using technology due to the health risks, addiction to technological products, the generation gap, safety issues, and social isolation [22]. Moreover, social interaction is mentioned as one of the main reasons or motivation for using technology for elderly people as they think that interacting with other people is crucial for their wellbeing [23]. It has been discovered that social interactions extend the social circles and help the elderly to meet new friends and make them easy to interact with the younger generation. Researchers mentioned that older people use technology to reduce their effort, to enhance their work, to cope with their needs and problems, and to compensate for their physical weakness [5]. Mahmood et al. [23] conducted a pilot study to explore the attitudes, preferences, and opinions of elderly people regarding the use of technology to extend and support their ability to “aging in place.” The results show that Safety and independence are also important factors for the elderly to use or nonuse of technology and they believe that the use of technology would significantly lead them to be safe and independent daily life [23]. Moreover, a qualitative study conducted to assess the usage of the patient portal by older patients with multiple chronic conditions shows that older people have the impression that usage of online portal saves time and money and give proper health information. The results also showed that older adults were more intent to use online portals because of the convenience of the health management system and perceived usefulness [21]. Literature also found that elderly people have a positive attitude towards mobile technology but they are also concerned about some complex functions, such as, age, attention, and capability of processing speed are critical factors that affected their usage [2]. Gaitán and colleagues reported that the technology usage behavior of elderly people is affected by habit, performance expectancy, price value, and effort expectancy [24]. Similarly, they highlighted some reasons for the non-use of technology by elderly people, such as; dispositional barriers, technological barriers, and situational barriers. For instance, forgetfulness is one of the dispositional barriers to the nonuse of technology by elderly people as they are easy to forget passwords of ATM etc. Health and ability conditions, like poor vision and hearing are also reported as the reasons for nonuse of technology [2]. Chen and Chan added the age related health and ability factors including; self-reported health conditions, functional and cognitive abilities and attitude to ageing and life satisfaction as the predictors of technology usage of elderly people [19]. Moreover, negative self-evaluated beliefs (too old to use technology), mental effort needed to operate advanced technologies, lack of interest, lack of time and assistance, limited access to and exposure to technology, expense, complexity, and safety are the reasons for nonuse of technology by elderly people mentioned by several studies [5, 19, 20, 25–28]. This suggests that use of e-health among elderly people is affected by several factors and generalizing them may not be the solution or compensation mechanism for all older people.

There are several technology acceptances models and theories that provided various factors predicting the usage, acceptance, and adoption of the technology by older people. In 1989, for the first time, Davis presented the technology acceptance model to predict who is more likely to accept the new technology, which was the adaptation of the two of the well-known theory of reasoned action presented by Fishbean and Ajzens in 1975, and the theory of planned behavior by Ajzan in 1991. The technology acceptance model is somehow the adaptation of the theory of reasoned action which states that beliefs determine the behavior intention of the user which determines the actual behavior. Hence, technology acceptance behavior is different from the theory of planned behavior as it states that the acceptance of technology is not solely dependent on the beliefs of the users. Venkatesh and Davis in 2000, extended the technology acceptance model known as TAM2, states that decision of the technology adoption depends on the outcome of the evaluation of the perceived ease of use (difficulty in using technology), their beliefs on perceived usefulness (using technology will increase their job performance), and subjective norms that state the influence of the people who are important to them [29]. In 2003, Venkatesh presented a new united theory of acceptance and use of technology (UTAUT), which identified three direct predictors of usage intention, i.e., performance expectancy, effort expectancy, and social influence, and two direct predictors of usage behavior (behavior intention and facilitating conditions), and also added four moderators as gender, age, experience, and voluntariness of use [30].

The purpose of the current research is to identify the list of the influencing indicators by using the Delphi method and to apply the multiple criteria decision analysis to prioritize the more or less potential barriers for the optimal solution to promote e-healthcare system usage among elderly people. We calculated priority weights of criteria and subcriteria by using AHP. the list of the main barriers and sub-barriers is compiled by the review of the previous literature shown in Table 1. Next, the research framework and results and findings are discussed in subsequent sections.

## 3. Research Framework and Methods

The framework in this study provides an insight for the healthcare providers and policymakers to closely observe and tackle the barriers to e-health usage. The research framework of our study is shown in Figure 1, where the DMAIC (define, measure, analyze, improve, and control) six sigma tool is used to design the checklist consisting of the potential barriers regarding the e-healthcare system usage. (DMAIC) is a data-driven strategy used to improve complex processes. This methodology is widely used in healthcare research [31–34].

There were five steps in DMAIC, the first step is to define. It is all about content validity which is done by reviewing the previous literature. The next step according to the DMAIC is the Measure “which means data collection here.” For our study, we used the Delphi method to collect the required data for this study. Delphi method is a widely used data collection technique in multiple criteria decision-making research [31, 35, 36]. This method provides a systematic way of getting the opinions from experts by using focused group discussions and questionnaires. The whole data collection was done in several steps. The data was collected by disseminating the checklist to 10 experts in March 2021 and getting the complete responses in April 2021. There was a total of 13 potential barriers in the checklist which were compiled in 3 major categories presented in Table 2. After identifying the potential barriers from the literature, the items were modified according to the Pakistani context. Then, the list was modified and verified by the group of experts again, to confirm whether the selected indicators are favorable in the Pakistani context or not.

The next step in the DMAIC was “Analyze and improve” the model. Multi-criteria decision analysis is a generalizable method for making decisions with dependencies and feedback [37]. Analytical hierarchy process (AHP) is a widely used technique in multiple criteria decision-making analysis, used by our study to analyze the e-healthcare barriers. This method has been used by researchers from diversified fields to simplify decision-making problems [38–42]. The detailed description of multiple criteria decision analysis and steps of the AHP method are explained in the next section. Finally, the last step in the DMAIC framework contains “control” which is all about concluding results, keeping them verified, committing to improvement, and passing along best recommendations to future researchers.

### 3.1. Data Collection

Past studies used a different number of experts to obtain reliable results for multiple criteria decision analysis; for example, Ikram et al. [43] used 10 experts to prioritize the barriers for integrated management assessment using the MCDM method. Whereas, another study used 4 experts for MCDM analysis to develop a model to choose an appropriate Computerized Maintenance Management System (CMMS) for a dairy company [44]. For the current research, 10 experienced experts were selected to rank the barriers and sub barriers. The participants were from academics from an aging research background, the healthcare sector, and policymakers. They were asked to prioritize the barriers based on their experts' opinions and experiences. All of the selected experts were having more than 10 years of experience, and have some research background in the aging care and e-healthcare management system.

### 3.2. Multiple Criteria Decision-Making (MCDM)

MCDM is a method of operational research that is commonly used to solve decision problems [45]. MCDM enables assessment and multiple expert judgments, and it is used to overcome the presence of imprecision and ambiguity during the evaluation process [46]. Several MCDM techniques have been discussed in the previous literature [37, 47]. However, each technique has unique characteristics and applications. The analytic hierarchy process (AHP) method of MCDM is used in this study to identify potential barriers to e-health use among the aging population.

#### 3.2.1. Analytical Hierarchical Process (AHP)

The AHP is a theory of measurement proposed by Saaty [13]. AHP is introduced to simplify the decision-making problems. AHP aims to compute relative priorities for a specified set of alternatives on a ratio scale which are centered on the decisions of experts, firmly following the consistency standard of pairwise comparison in the process of decision-making [48]. The strong point of this method is that it provides a structured yet relatively simple solution and organizes tangible and intangible factors in a logical way to the decision-making problems (Shen & Li, 2005). In this study, the Analytical hierarchy process (AHP) is used to identify e-healthcare barriers. This method is used because of its unique utilization of a hierarchy structure to represent a problem in the form of a goal, criteria, and alternatives [13]. AHP's main components are pairwise comparisons, developing and comparing matrices, and ensuring their consistency. This technique assists all decision-makers in selecting and ranking complex problems rationally. The following steps are involved in the computations of this method:

*(1) Step-I: Constructing Hierarchy*. First of all, the problem has to be structured into hierarchies with different layers defined as a goal, criteria, and alternatives. The goal is the main purpose of constructing the model. The second level of the hierarchy must be composed of some criteria based on which the researcher is going to evaluate the alternatives. The third important part or layer of hierarchy is the alternatives or the main areas of evaluation. The respondents have to be selecting the alternatives based on the given criteria. The hierarchy can consist of many sub-criteria and alternatives. According to Saaty, the criteria for each dimension should be mutually independent [13].

*(2) Step-II: Deriving Weights or Priorities for the Criteria*. The next step is to perform a pairwise comparison of the respondents' or experts' judgments to determine the comparative weights. This step yields the ranked priorities for the alternatives under each criterion. Based on a standard evaluation scheme, Saaty developed a scale for pairwise comparisons. In this step, the components of a certain level are compared with respect to a specific component in the direct upper level. The consequential weights of the components may be referred to as local weights.

*(3) Step-III: Calculating Priorities*. The judgment matrices are then used to calculate the priorities. The Eigenvalue method is the method most commonly used by researchers for this step [49–51].

*(4) Step-IV: Model synthesis or Final Ranking*. In this step, the calculated priorities are combined or aggregated as a weighted sum to establish or obtain the overall ranking of the best alternative.

*(5) Step-V: Consistency*. After getting the results, it is required to check the consistency to verify the model. The Saaty introduced the threshold of 10% or 0.01 as the acceptable inconsistencies in the data. AHP computes the consistency ratio (CR), by comparing the consistency index (CI) of the matrix in question (with our evaluations) with the consistency index of a random matrix (RI). The formula for the consistency check is given by Saaty as

(1) $$\begin{array}{c} \text{CR}=\frac{\text{CI}}{\text{RI}}, \end{array}$$

where

(2) $$\begin{array}{c} \text{CI}=\frac{\lambda_{\max}-n}{n-1}. \end{array}$$

Here CI represents consistency index, and CR as consistency ratio, *λ*_max_ represents the biggest eigenvalue of the pair-wise comparison matrix, *n* is the matrix order, and RI is a random index. If the value of CR is less than 10% then the matrix is considered as having an acceptable consistency. In some cases, 20% can also be acceptable but not more [13]. If the CR does not lie within the given threshold or acceptable range then decision-makers have to be revised their judgments.

## 4. Results and Discussion

This study aims to identify barriers to the use of the e-healthcare system by elderly people, to better facilitate the future development of a digital healthcare system for the aging population. The AHP method was used to calculate the weights by using a geometric mean. We used the group-based decision-making approach to calculate the weights for the e-healthcare barriers and sub-barriers. For the MCDM analysis, we categorized sub-barriers into three main barriers, i.e., Attitudinal barriers, socio-environmental barriers, and health and ability barriers. The weights were calculated for the 3 main barriers first and then for the sub-barriers.  Figure 2, shows the hierarchal structure of e-healthcare barriers and sub-barriers. Table 2 shows the results of the AHP method.

### 4.1. Main Barriers

The weights of each main barrier were calculated by using the AHP technique. The results in Figure 3, show that ‘Health and ability' are resulted to be the most potential barrier weighting (0.6334), followed by socio-environmental (0.2604), and attitudinal barrier (0.1061), respectively. These barriers seem to be a challenge for implementing the e-healthcare system for the aging population. Sound health and ability constructs are the foremost barriers highlighted to be addressed to ensure the effective use of e-health among older adults. Manufacturers, policymakers, and healthcare providers should focus on age-related health problems while framing and implementing the e-healthcare technology. Socio-environmental and attitudinal barriers are placed at second and third priorities by the experts. To facilitate e-health use among the aging population, the manufacturers and policymakers should carefully prioritize the barriers as per their potential strengths and weaknesses. E-healthcare manufacturers should design the products in a manner that can overcome the barriers and construct an elderly user-friendly e-health technology system for more optimal outcomes while considering these potential barriers. Gerontechnologies should manufacture to facilitate the users without facing any challenges. There is a need to accept the age-specific requirements to better implement the use and to facilitate the e-health care system for elderly people. Finally, attitudinal characteristics are turned out as the least important barrier, revealing that the use of e-health can be impacted by attitudinal beliefs but with less intensity. Additionally, the 14 sub-barriers were assessed by using a pairwise comparisons matrix.

### 4.2. Sub-barriers

The detailed results of the sub-barriers are given as follows.

#### 4.2.1. Attitudinal Sub-Barriers

The Attitudinal sub-barriers are ranked as follows:

(3) $$\begin{array}{c} \text{AD}-14>\text{AD}-13>\text{AD}-12>\text{AD}-11. \end{array}$$

Negative attitude towards life and life satisfaction appeared as the most potential sub-barrier (AD-14) of attitudinal barrier with a weight of (0.53). This ranking represents the reality that lack of life satisfaction leads older adults towards isolation and increase depression and feeling of social withdrawn. Such feelings may lead older towards the lack of interest in technology and e-health system. The positive life satisfaction in older age depends on multiple factors, such as poverty, lack of income, poor health, and depression, as mentioned in a previous study [45, 52]. The second sub-barrier is the lack of perceived ease of use among older adults (AD-13) with 0.2314 priority weight. Perceived ease of use is defined as “the degree to which a person believes that using a technology will be free from effort” (p.320). Previous studies maintained that perceived ease is strongly associated with the use of technology among older adults [21, 53]. User-friendly and effort-free e-healthcare products encourage the use of e-health among older adults. Moreover, perceived usefulness is resulted to be the third influential sub-barrier (AD-12) under the category of attitudinal barrier with a weight of (0.1725). Perceived usefulness is defined as “the extent to which a person believes that using a particular technology will enhance his/her job performance” [54]. factors affecting technology usage among older adults within the literature focus on the importance of attitudinal factors, whereas some studies revealed that there is no significant effect of Perceived usefulness on the technology usage behavior of older adults [19, 20]. Further, a negative attitude towards using technology has appeared as the least important sub-barrier (AD-11, 0.0688) of the Attitudinal barrier. Attitude towards using technology is mainly used as a dependent variable in the previous studies, influence by several other factors [21]. A positive attitude towards technology motivates the elderly to accept and use e-health technology. Results are displayed in Figure 4.

#### 4.2.2. Socio-Environmental Sub-Barriers

The ranking of the sub-barriers under the category of socio-environmental barrier is as follows:

(4) $$\begin{array}{c} \text{SE}-24>\text{SE}-23>\text{SE}-21>\text{SE}-22. \end{array}$$

Insufficient funds (0.5666) have resulted as the greatest challenge for elderly people to use e-healthcare technology. The findings show that the cost of e-health for the aging population should be economical for better health outcomes. Therefore, sufficient funds or cost tolerance would increase the use of e-health among elderly and the facilitate the smart health care agenda of policymakers. Several studies have considered the importance of the financial status, occupation, and income, that may influence the technology usage behavior of elderly people [20, 55, 56]. Pakistan is a developing country and per capita income is relatively low as compared with other developed countries [57], especially older people who have a low socio-economic background and are concerned with the costs of technological products and services. Hence, we may assume that Cost tolerance is a significant predictor of e-health usage behavior of elderly people.

Lack of social support is prioritized as the second potential sub-barrier (SE-23, 0.2477) under this category. Elderly people who suffer from social exclusion and lack of social support from friends and family may have the least interest in using e-health which affects their healthcare access. A previous study also mentioned social interaction as the motivation for using technology for elderly people as they think that interacting with other people is crucial for their wellbeing [23].

Insufficient facilitating conditions are prioritized as the third potential (SE-21, 0.0986) sub-barrier under the category of the socio-environmental barrier. Facilitating conditions are the environmental factors that support the usage of technology by elderly people. Venketesh in 2003, presented a united theory of technology acceptance (UTAUT) and found the facilitating conditions as a direct predictor of technology usage behavior [30]. A study in India about the ICT usage behavior of elderly people revealed that facilitating conditions are positively associated with technology usage [58]. Hence, a lack of facilitating conditions may affect the successful promotion of e-health use.

The last sub-barrier under the socio-environmental barrier is the negative subjective norm (SE-22) with (0.0922). Subjective norm is defined here as the influence of the people who are important to the elderly [29]. Negative influence from peers and family may hinder access to e-health usage and result in poor health care [59]. See Figure 5.

#### 4.2.3. Health and Ability Barriers

Figure 6 shows the results of sub-barriers under the category of health and ability barriers with the results as follows:

(5) $$\begin{array}{c} \text{HA}-35>\text{HA}-34>\text{HA}-32>\text{HA}-33>\text{HA}-31. \end{array}$$

Based on the expert's opinion, anxiety is prioritized as the most potential sub-barrier (HA-35) with weight (0.4833). Anxiety is defined as the individual hesitation when he or she intends to use the system [60]. Chen and Chan used anxiety in their senior technology acceptance model and the results show that anxiety has a negative influence on the technology usage behavior of elderly people [20]. Hence, the proper guidelines and understanding of the healthcare system may help elderly people to reduce anxiety and increase their motivation towards the effective use of the e-health system. Furthermore, self-efficacy has resulted as a second potential sub-barrier (HA-34, 0.2509) under the health and ability barriers. Self-efficacy is generally defined as the person's judgment of his or her ability to use the system [45]. It has been declared as a potential factor in previous studies which affects the use of technology among older adults [20]. Lack of cognitive ability is prioritized as the third sub-barrier (HA-33) in this category with the weight of (0.1046). A previous study stated the importance of cognitive abilities for older adults in using technology [14]. The difference between (HA-33) and (HA-32) weights is 0.0031, which shows their almost equal importance for e-healthcare use among elderly people. psychological health factors are positively affecting the technology usage behavior of older people [19]. The last sub-barrier under this category is physical health with (0.0535) weight, showing its least importance in the use of e-health system.

### 4.3. The Overall Ranking of Sub-Barriers

Figure 7, shows the overall ranking of all the sub-barriers by calculating the final weights of all sub-barriers. The calculations are done by using the weight of each sub-barrier and multiplying it by the weight of its respective main barrier. The results of the ranking of overall sub-barriers are as follows:

(6) $$\begin{array}{c} \text{HA}-35>\text{HE}34>\text{SE}-24>\text{HA}32>\text{HE}-33>\text{SE}-23>\text{AD}-14>\text{HA}-31>\text{SE}-21>\text{AD}-13>\text{SE}-22>\text{AD}-12>\text{AD}-11\text{.} \end{array}$$

Anxiety is resulted to be the ranked first potential sub-barrier with the weight (0.306) among all other, followed by self-efficacy (0.159), insufficient funds (0.148), and lack of psychological fitness (0.068). The least three sub-barriers have resulted as a negative subjective norm (0.024), lack of perceived usefulness (0.018), and negative attitude towards technology (0.007) respectively.

## 5. Conclusion

The need for tools that aid in decision-making occurs in a variety of healthcare settings and these tools are employed to varying degrees in different settings [61]. In this study, we focus on the possibilities of using a specific multiple criteria decision-making technique in ranking potential barriers for e-health use among elderly people. The findings show that health and ability constructs are crucial to address while encouraging the use of e-health system for elderly people. Our findings are vital to decision makers in the field of geriatrics and healthcare technology to focus on the age related health and ability characteristics while introducing any innovation in an e-health system.

Since the identification of the potential barriers and sub-barriers is an innately complex system that cannot be represented using a single metric only, multidimensional (MCDA) approaches are highly suggested to identify potential risks. Hence, our study aimed to investigate the feasibility of employing the AHP approach to identify possible barriers to e-health use among older adults. The technique presented in this paper is quite simple. Any spreadsheet may be used to execute mathematical operations, which is very important for small sample sizes. The AHP technique may be successfully utilized in the healthcare domain to analyze, compare, and identify the potential barriers, and to prioritize them according to their worst scenarios, as shown in the studies and analyses presented here. Utilizing the MCDA techniques in the present study will assist the public health practitioners and policymakers in drawing decisions on the best way to minimize the risks in the e-health system that plays a significant role in facilitating the smart health care industry for the aging population. More importantly, this investigation facilitates researchers with an MCDA roadmap to help them enhance the quality of their studies and their understanding of how to use MCDA techniques to evaluate and prioritize the influencing factors affecting e-health use in healthcare research.

## Figures and Tables

**Figure 1:** Research framework operationalized in the study.

**Figure 2:** Hierarchical structure of e-health management system barriers.

**Figure 3:** Ranking of main barriers based on AHP.

**Figure 4:** The ranking order of attitudinal sub-barriers.

**Figure 5:** The ranking of socio-environmental sub-barriers.

**Figure 6:** The ranking of health and ability sub-barriers.

**Figure 7:** The overall ranking of sub-barriers.

**Table 1:** Potential barriers to e-health usage system for the aging population.

Main barriers	Sub-barriers	References
Attitudinal (AD-1)	Negative attitude towards using technology (AD-11)	[19–21, 24, 28]
	Lack of perceived usefulness (AD-12)	
	Lack of perceived Ease of use (AD-13)	
	Negative attitude towards life and life satisfaction (AD-14)	
Socio-Environmental (SE-2)	Insufficient facilitating conditions (SE-21)	[23, 24, 30]
	Negative subjective norm (SE-22)	
	Lack of social support (SE-23)	
	Insufficient funds/Cost Tolerance (SE-24)	
Health and Ability (HA-3)	Physical health (HA-31)	[2, 22] [5, 19, 20]
	Lack of psychological fitness (HA-32)	
	Lack of cognitive ability (HE-33)	
	Lack of self-efficacy (HA-34)	
	Suffering from anxiety (HA-35)	

**Table 2:** Estimated AHP weights for main and sub-barriers.

Main barriers	Main barriers weights	Sub-barriers code	Consistency ratio (CR)	Priority weight	Final weight
Attitudinal (AD-1)	0.1061	AD-11	0.03	0.0688	0.007
		AD-12		0.1725	0.018
		AD-13		0.2314	0.025
		AD-14		0.5357	0.057
Socio-Environmental (SE-2)	0.2604	SE-21	0.03	0.0986	0.026
		SE-22		0.0922	0.024
		SE-23		0.2477	0.065
		SE-24		0.5666	0.148
Health and Ability (HA-3)	0.6334	HA-31	0.01	0.0535	0.034
		HA-32		0.1077	0.068
		HA-33		0.1046	0.066
		HA-34		0.2509	0.159
		HA-35		0.4833	0.306

## Data Availability

The data used to support the findings of this study are available from the corresponding author upon request.
